# A combination of intradermal jet-injection and electroporation overcomes *in vivo* dose restriction of DNA vaccines

**DOI:** 10.1186/1479-0556-10-5

**Published:** 2012-08-08

**Authors:** David Hallengärd, Andreas Bråve, Maria Isaguliants, Pontus Blomberg, Jenny Enger, Richard Stout, Alan King, Britta Wahren

**Affiliations:** 1 Department of Microbiology, Tumor and Cell Biology, Karolinska Institute, Nobels väg 16, 171 77, Stockholm, Sweden; 2 Swedish Institute for Communicable Disease Control, Nobels väg 18, 171 82, Solna, Sweden; 3 Vecura, Karolinska University Hospital, 141 86, Huddinge, Sweden; 4 Bioject Medical Technologies, 7180 SW Sandburg St, Tigard, Oregon, 97223, USA; 5 Cellectis, 102 avenue Gaston Roussel, Romainville, France

**Keywords:** DNA vaccine, Electroporation, Jet-injection, Biojector

## Abstract

**Background:**

The use of optimized delivery devices has been shown to enhance the potency of DNA vaccines. However, further optimization of DNA vaccine delivery is needed for this vaccine modality to ultimately be efficacious in humans.

**Methods:**

Herein we evaluated antigen expression and immunogenicity after intradermal delivery of different doses of DNA vaccines by needle or by the Biojector jet-injection device, with or without the addition of electroporation (EP).

**Results:**

Neither needle injection augmented by EP nor Biojector alone could induce higher magnitudes of immune responses after immunizations with a high dose of DNA. After division of a defined DNA dose into multiple skin sites, the humoral response was particularly enhanced by Biojector while cellular responses were particularly enhanced by EP. Furthermore, a close correlation between* in vivo* antigen expression and cell-mediated as well as humoral immune responses was observed.

**Conclusions:**

These results show that two optimized DNA vaccine delivery devices can act together to overcome dose restrictions of plasmid DNA vaccines.

## Background

Plasmid-based DNA vaccines are commonly used in vaccine research to induce immune responses against infectious agents or tumor antigens. These vaccines possess advantages including rapid construction and high stability, as well as the capacity to induce cellular immune responses owing to the intracellular production of the encoded antigen [1]. Still, further optimization of DNA vaccine delivery is needed for this vaccine modality to ultimately be efficacious in humans [2,3].

One strategy to influence the immune responses to DNA vaccines is by the choice of immunization route. We have chosen to employ intradermal (id) immunizations as the skin, unlike muscle tissue, has a large population of resident antigen presenting cells (APCs) that can facilitate the induction of vaccine-specific immune responses [4,5]. The skin is also a more accessible tissue than muscle, allowing for less painful DNA vaccine delivery and facilitating studies of *in vivo* protein expression. In addition to conventional needle immunization, several injection devices including Biojector and *in vivo* electroporation (EP) are being used to improve DNA delivery to the skin. Biojector is a CO_2_-propelled needle-free device that injects DNA plasmids as a highly focused liquid stream into the skin. This has been shown to enhance antigen expression as compared to conventional needle injection [6], most probably due to the large area and thus larger number of cells being targeted by injection with Biojector. DNA vaccine delivery by Biojector has been shown to induce strong immune responses in preclinical and clinical trials [6-11].

Another commonly used strategy employed to augment DNA vaccine delivery is EP. EP enhances transfection efficacy by the transient formation of pores in the cell membrane, allowing for an increased uptake of plasmids into the cell. Additionally, the electric pulses result in an influx of APCs to the site of injection [12,13], further augmenting the immunogenicity of the gene product. Thus, EP can significantly enhance expression [13,14] and immunogenicity [15-18] of plasmid-encoded antigens.

Similar to other vaccine modalities, the DNA vaccine dose influences immunogenicity, and immune responses are generally enhanced by increasing the dose [12,19-22]. Still, an upper limit in terms of *in vivo* expression [23-26] and immunogenicity [27,28] has been observed in mice after intramuscular (im) and id injections. This plateau appears at doses of 5–100 μg DNA delivered at concentrations ranging between 0.3-2 μg/μl. Limitations in cellular uptake of plasmids and clearance of antigen expressing cells by immune cells [29-33] have been suggested to account for this phenomenon. One way to override this issue is by dividing the plasmid dose at several injection sites rather than a single location [9-11,25,28]. Using too many injections may however limit the feasibility, making plasmid vaccines less attractive for use in the clinic. It has also been shown that protein expression can be enhanced when increasing the plasmid concentration [34,35], suggesting that an increase in plasmid concentration can be an alternative to large volumes and multiple injections of DNA vaccines.

In this study we evaluated the capacity of different id DNA immunization strategies to induce immune responses in mice. DNA was delivered by needle or Biojector, with or without the addition of EP. Luciferase- and HIV-1 Gag-encoding plasmids of various concentrations were used in order to determine the impact of DNA dose on *in vivo* expression and immunogenicity in mice, respectively. To avoid dose limitations by volume restrictions when delivering DNA vaccines id, we used plasmid preparations of up to 10 μg/μl. The study showed that a high dose of DNA injected by Biojector alone (1000 μg) or needle plus EP (100 μg) induced similar levels of immune responses as a considerably lower dose of DNA (10 μg) administered in the same manner. Interestingly, when we combined Biojector-injection with EP, this dose plateau could be circumvented as evidenced by the significantly stronger immune responses that were induced after immunization with the high dose DNA as compared to the lower dose. Furthermore, a close correlation between the level of *in vivo* antigen expression and frequency of cell-mediated immune responses, and between reduction in *in vivo* antigen expression and magnitude of CD8^+^ T cell responses, were observed. These data suggest that a combination of Biojector and EP could overcome dose restrictions observed also for other DNA encoded antigens.

## Methods

### Vaccine formulation and immunizations

pKCMVp37B [10,36], pVax-Luc [13] and empty pKCMV were used for immunizations. Plasmids were amplified in *E. Coli* and purified using endotoxin-free GigaPrep (QIAGEN, Hilden, Germany) and PlasmidSelect (GE Healthcare) kit. The eluted and precipitated DNA was dissolved in saline at 4°C overnight to obtain DNA of 10 μg/μl. Gel-clot tests for detecting endotoxins in DNA preparations were performed at APL Pharma Specials (Stockholm, Sweden).

Female BALB/c mice (Charles River Laboratories, Sülzfeld, Germany), 5–8 weeks old, were held at the Astrid Fagraeus Laboratory (Ethical approval Dnr: N210/07). Mice were immunized once or twice (week 0 and 4) id on the back of the mouse. Doses of 10–1000 μg DNA were injected with a 29 gauge Micro-Fine™ needle (BD, NJ, USA) or by Biojector [10] (Bioject Medical Technologies, OR, USA) with dermal spacer, with 10 and 100 μl DNA solutions diluted in saline, respectively. The Biojector was adjusted for delivery to mice (3400 PSI). Immunizations with needle and Biojector were either given alone or followed by EP using the Derma Vax™ EP device (Cellectis, Romainville, France) as previously described [13]. Briefly, the needle electrodes (2 mm) were inserted in the shaved mouse skin to cover the injection site and two pulses of 1125 V/cm (50 μs duration) plus eight pulses of 275 V/cm (10 ms duration) were applied.

### Cellular immune responses

Mice were sacrificed two weeks after the last immunization or, for the *in vivo* imaging study, 25 days after a single immunization, and spleens and serum were collected. Splenocytes were purified by Ficoll-Paque separation (GE Healthcare, Stockholm, Sweden) and IFN-γ ELISpot and IFN-γ/IL-2 FluoroSpot assays (Mabtech, Nacka Strand, Sweden) were performed according to the manufacturer’s protocol and as previously described [37]. 1 × 10^5^ viable cells were plated per well and stimulated with a peptide pool covering Gag p24B (15mers with ten amino acids overlap) or the H2-K^d^ restricted AMQMLKETI (Gag) and GFQSMYTFV (luciferase) [38] peptides. The final concentration of peptides was 5 μg/peptide/ml.

### Antibody responses

Binding antibody titers were assessed with ELISA as previously described [39]. Plates were coated with 100 μl/well of 1 μg/ml recombinant Gag p17/p24B (NIBSC/CFAR, Potters Bar, UK) or recombinant luciferase (Promega, WI, USA).

### *In vivo* expression

Subsequent to DNA injections, mice were injected intraperitoneally (ip) with luciferin potassium salt (Caliper Life Sciences, MA, USA) and luciferase expression was assessed by using the IVIS200 apparatus (Xenogen, CA, USA) as previously described [13]. In the present study*, in vivo* expression was assessed ten minutes after ip injection with luciferin and injections with different doses of pVax-Luc and pKCMVp37B were compared with the corresponding dose of empty pKCMV plasmid.

### Statistical analysis

Statistical analysis was performed using the GraphPad Prism 4 software (GraphPad Software, CA, USA). A two-tailed Mann–Whitney test and a Spearman rank test were used to analyze differences between two groups and correlation between *in vivo* expression and immunogenicity.

## Results and discussion

### High and low plasmid dose administered by Biojector or needle followed by EP induce similar levels of immune responses

The first study was designed to compare id vaccine delivery by Biojector with id needle injections augmented by EP, and evaluate whether a high dose vaccine plasmid (1000 μg for Biojector and 100 μg for needle plus EP), delivered either as single or multiple injections, could induce stronger immune responses than a considerably lower dose (10 μg). Hence, BALB/c mice were immunized twice with different doses and volumes of a HIV-1 Gag-encoding plasmid (pKCMVp37B) [10,36], either by Biojector or with needle followed by EP.

Although we used a larger volume and thus higher plasmid dose when immunizing with Biojector (100 μl), than when immunizing with needle and EP (10 μl), needle and EP induced higher magnitudes of IFN-γ secretion when the DNA was delivered at multiple injection sites and stronger antibody responses for both high and low vaccine doses (p < 0.05) (Figure 1). This suggests that EP is superior to Biojector to augment the immunogenicity of plasmid vaccines.

**Figure 1:** **Impact of DNA vaccine dose and id delivery devices on immunogenicity.** BALB/c mice were immunized week 0 and 4 with pKCMVp37B with either Biojector (BJ) or with needle followed by electroporation (EP). For Biojector, 10, 5 × 200 or 1000 μg DNA was delivered in 100 μl saline/injection. For needle plus EP, 10, 5 × 20 or 100 μg was delivered in 10 μl saline/injection. **A)** Cellular immune responses were assessed by IFN-γ ELISpot on splenocytes collected two weeks after the second immunization. A peptide pool representing Gag p24B was used to stimulate splenocytes. **B)** Binding antibodies to Gagp17/p24B were addressed by ELISA on serum collected two weeks post the last immunization. Bars represent mean values. *Significant difference (p < 0.05). ns = no significant difference.

In terms of DNA dose, both Biojector and needle plus EP immunized mice mounted similar magnitudes of immune responses after immunization with the high (1000 μg for Biojector and 100 μg for needle plus EP) and the low (10 μg) dose (Figure 1). These results suggest that a dose plateau was reached prior to or at the low dose, that prevented further amplification of immune responses, despite the use of two powerful DNA delivery devices. No endotoxins were detected in neither of the DNA preparations. Hence, we could exclude that traces of endotoxins in the highly concentrated DNA preparations (10 μg/μl) accounted for the limited immune response that was induced in mice immunized with the high dose DNA.

The limited cellular and humoral immune responses induced by a high dose of DNA in both Biojector and needle plus EP immunized mice appeared somewhat elevated (p > 0.05) when the total amount of DNA was divided and delivered as five injections on different injection sites (5 × 200 μg for Biojector and 5 × 20 μg for needle plus EP). Mice immunized with Biojector even displayed significantly improved binding antibody titers (p < 0.05). The superiority of multiple-site immunizations has previously been observed after im needle immunizations [28], and after id needle plus EP immunizations [25]. Here we demonstrate that this phenomenon applies also for antibody responses after plasmid vaccine delivery with Biojector.

### The addition of EP enhances immune responses of needle and Biojector immunizations

As neither delivery by Biojector nor needle plus EP could circumvent the observed dose plateau and elicit stronger immune responses after immunizations with a high dose of DNA as compared to a low dose, the combined effect of Biojector and EP was studied. BALB/c mice were immunized twice with 10 μg pKCMVp37B by needle (10 μg in 10 μl) or Biojector (10 μg in 100 μl), with or without the addition of EP.

The results showed that needle and Biojector delivery, with or without the addition of EP, induced similar levels of IFN-γ and Gag-specific antibody titers (Figure 2). The addition of EP to needle and Biojector immunizations however enhanced the IFN-γ responses for both modes of vaccine delivery, and antibody responses for needle plus EP delivery (p < 0.05). Hence, although Biojector has been shown to induce strong immune responses to DNA vaccines, we show that when immunizing with a low dose DNA, with or without the addition of EP, Biojector does not induce stronger immune responses than conventional needle delivery. Similar observations have been reported when comparing the efficacy of needle and Biojector DNA vaccine delivery id in pigs [6], or im in cynomolgus monkeys [40]. However, a more concentrated DNA has been reported to correlate with stronger immune responses [34,35]. The inability of Biojector immunizations to induce stronger immune responses than needle immunizations might thus be explained by the more diluted DNA being injected by Biojector, as 100 μl is the smallest volume that can be delivered by this device.

**Figure 2:** **Immune responses induced by different means of id DNA vaccine delivery.** 10 μg pKCMVp37B was diluted in 10 or 100 μl saline and delivered by needle or Biojector (BJ), respectively. Also mice immunized with needle or Biojector followed by electroporation (EP) were included. Immunizations were done week 0 and 4. **A)** Cellular immune responses were assessed with IFN-γ ELISpot on splenocytes collected two weeks after the second immunization. A peptide pool representing Gag p24B was used to stimulate splenocytes. **B)** Gag-specific IgG titers in serum collected at the same time point were determined by Gagp17/p24B ELISA. Bars represent mean values. *Significant difference (p < 0.05) and **significant difference (p < 0.01). ns = no significant difference.

### Injections with high DNA doses by a combination of Biojector and EP induce luciferase-specific cell-mediated immune responses

To further evaluate the combined effect of Biojector and EP, we studied *in vivo* protein expression after Biojector plus EP injections. BALB/c mice were immunized once with doses ranging from 10 to 1000 μg of a luciferase-encoding plasmid (pVax-Luc) [13] or empty vector (pKCMV). Subsequent luciferase expression *in vivo* was measured using the Xenogen *In Vivo* Imaging System (IVIS), which allows for a direct quantification of luciferase expression visualized as luminescent pixels after cleavage of an ip injected luciferin substrate. Expression was measured at 4, 8, 11, 18 and 25 days post injection and immune responses were assessed by ELISA and IFN-γ/interleukin-2 (IL-2) FluoroSpot [37] at day 25.

There was a decrease in luciferase expression at the later time points in mice being injected with large doses of DNA, as compared to mice receiving the low doses (Figure 3A). Luciferase has been reported to be weakly immunogenic [33,41] and Limberis *et al.* identified murine CD8^+^ T cell epitopes in luciferase [38]. Thus, the dominant H2-K^d^ restricted GFQSMYTFV epitope was used in this study to establish whether any luciferase-specific CD8^+^ T cell responses were induced. The highest dose Luciferase-encoding plasmid induced higher IFN-γ, IL-2 and IFN-γ/IL-2 responses than the lowest dose (p = 0.03) (Figure 3B), and the level of antigen expression at day 8 correlated with the magnitude of cell-mediated immune responses (p < 0.05) (Figure 3C). Furthermore, the level of CD8^+^ T cell responses commonly correlate with the ability of these T cells to clear transfected cells [29,33,42]. The increased CD8^+^ T cell responses did, however, not correlate with the decreased luciferase-expression observed in Figure 3A (data not shown), perhaps due to the limited levels of IFN-γ and IL-2 responses induced even in the high dose group. No luciferase-specific antibody responses were induced in any of the groups (data not shown).

**Figure 3:** ***In vivo *luciferase expression following Biojector plus EP injections with escalating doses of DNA.** BALB/c mice were immunized once with Biojector followed by EP with 10-1000 μg of a luciferase-encoding plasmid (pVax-Luc) or empty vector diluted in 100 μl saline. **A)** 4, 8, 11, 18 and 25 days post DNA injections mice were injected ip with the D-luciferin substrate and expression of luciferase was monitored using the Xenogen *In Vivo* Imaging System (IVIS). Results are shown as mean values (n = 4) and error bars represent standard error of the mean. **B)** At day 25, spleens were collected and IFN-γ, IL-2 and IFN-γ/IL-2 responses were assessed by FluoroSpot. The H2-K^d^ restricted GFQSMYTFV (luciferase) and AMQMLKETI (Gag) peptides were used to assess luciferase-specific and unspecific cytokine secretion, respectively. Bars represent mean values for the GFQSMYTFV peptide. **C)** Correlation between *in vivo* expression at day 8 and frequency of GFQSMYTFV-specific IFN-γ, IL-2 and IFN-γ/IL-2 secreting splenocytes at day 25. *Significant difference (p < 0.05).

### Immunizations with a combination of Biojector and EP overcome dose restrictions to plasmid-encoded Gag

We next examined how the Biojector plus EP immunization strategy with different doses applied for the Gag-encoding DNA that was used in the two initial experiments. BALB/c mice were immunized once with doses ranging from 10 to 1000 μg of pKCMVp37B or empty vector (pKCMV), both mixed with 25 μg pVax-Luc to examine the *in vivo* immunogenicity measured as the clearance of pKCMVp37B and pVax-Luc transfected cells. The 25 μg pVax-Luc dose was chosen as it does not induce luciferase-specific immune responses (Figures 3A and B).

The initial level of luciferase expression did not differ significantly between groups (Figure 4A). An increase in dose of pKCMVp37B was however associated with a more rapid decline of luminescence. Results from the FluoroSpot assay demonstrated that the mice receiving the highest dose of Gag-encoding plasmid obtained significantly stronger IFN-γ responses than mice immunized with the lowest dose (p < 0.03) (Figure 4B). A strong negative correlation between the frequency of IFN-γ, IL-2 and IFN-γ/IL-2 responses and level of luciferase expression was seen at 25 days post immunization (p < 0.01) (Figure 4C), indicating that Gag-specific immune responses can clear cells co-transfected with Gag- and luciferase-encoding plasmids, and perhaps bystander cells transfected with luciferase-encoding plasmids only [43]. In addition, immunizations with the high doses of Gag-encoding plasmid led to a more rapid and enhanced reduction in luminescence than injections with high doses of luciferase-encoding plasmid (Figure 3A and Figure 4A), showing that Gag is more immunogenic than luciferase. This was also seen in the FluoroSpot assays (Figure 3B and Figure 4B).

**Figure 4:** **Immunogenicity of Gag following Biojector plus EP immunizations with escalating doses of DNA.** BALB/c mice were immunized once with Biojector followed by EP with mixtures of 10–1000 μg pKCMVp37B or empty vector and 25 μg pVax-Luc diluted in 100 μl saline. **A)** 4, 8, 11, 18 and 25 days post DNA injections mice were injected ip with the D-luciferin substrate and expression of luciferase was monitored using the Xenogen *In Vivo* Imaging System (IVIS). Results are shown as mean values (n = 4) and error bars represent standard error of the mean. **B)** At day 25, spleens were collected and IFN-γ, IL-2 and IFN-γ/IL-2 responses were assessed by FluoroSpot. A Gag p24B peptide pool was used to assess Gag-specific cellular immune responses, and the H2-K^d^ restricted GFQSMYTFV (luciferase) peptide was used to assess luciferase-specific responses. Bars represent mean values for the Gag p24B peptide pool. **C)** Correlation between *in vivo* expression and frequency of Gag p24B peptide pool-specific IFN-γ, IL-2 and IFN-γ/IL-2 secreting splenocytes at day 25. **D)** Antibody titers to Gag p17/p24B were assessed by ELISA on serum collected 25 days post immunization. Bars represent mean values. *Significant difference (p < 0.05).

Similar to the two initial studies with pKCMVp37B, the Gag p24B peptide pool and the H2-K^d^ restricted AMQMLKETI peptide stimulated comparable levels of cellular immune responses in the ELISpot and FluoroSpot assays (p < 0.05 for all groups) (data not shown), demonstrating that the induced cell-mediated immune responses, including those responsible for the clearance of Gag-expressing cells, are mainly of CD8^+^ T cell nature. With respect to antibody responses, the titers of Gag-specific binding antibodies were enhanced as the dose of Gag-encoding plasmid was increased, and the mice receiving the highest dose elicited significantly higher antibody titers than mice immunized with the lowest dose (p = 0.03) (Figure 4D).

Biojector plus EP immunizations have previously been studied in pigs [6]. That study showed that a combination of Biojector and EP lead to a more rapid induction of antibody responses as compared to needle plus EP delivery. However, there was no difference in the magnitude of antibody titers. Here we demonstrate that the combination of Biojector and EP can overcome the observed dose restriction of a Gag-encoding plasmid and enhance immune responses when the DNA vaccine dose is increased. This is most probably a consequence of enhanced transfection efficacy of id delivery, in part by targeting a large number of cells with Biojector, and in part by improved cellular uptake when adding EP. We assume that the observed antigen expression and subsequent immune response indeed are located in the dermal layer of the skin and not in underlying muscle since we use a Biojector device that is adjusted for id delivery to mice. Moreover, we have previously shown that approximately 1000-fold less DNA is located in the underlying muscle as compared to the injected skin after Biojector plus EP immunizations in mice [44].

## Conclusions

In summary, the present findings demonstrate that the combination of Biojector and EP can overcome the observed dose restriction of a DNA vaccine and enhance immune responses when the dose is increased. Furthermore, we show that levels of antigen expression correlate with the frequency of IFN-γ and IL-2 secretion, and that the clearance of antigen expression correlates with the magnitude of IFN-γ responses to CD8^+^ T cell epitopes. Although the high concentration and thus high doses of DNA used in this study are too high to translate directly into human settings, these comparisons show that these two modes of optimized DNA vaccine delivery can act together to overcome dose restriction of a plasmid DNA vaccine.

## Competing interests

RS and AK are employees at Bioject Medical Technologies and Cellectis Bioresearch, respectively.

## Authors’ contributions

DH performed the experiments and drafted the manuscript. All the authors read and approved the final manuscript.
